The article "Investigation of Metastasis-Related Genes: A Rat Model Mimicking Liver Metastasis of Colorectal Carcinoma" was published in 2017. Journal: Front Oncol.

# Investigation of Metastasis-Related Genes: A Rat Model Mimicking Liver Metastasis of Colorectal Carcinoma

**DOI:** 10.3389/fonc.2017.00152

**Published:** 2017-07-18

**Authors:** Hassan Adwan, Rania Georges, Asim Pervaiz, Martin R. Berger

**Affiliations:** ^1^Faculty of Pharmacy and Biotechnology, Department of Pharmacology and Toxicology, The German University in Cairo, Cairo, Egypt; ^2^Toxicology and Chemotherapy Unit, German Cancer Research Center, Heidelberg, Germany; ^3^Department of Allied Health Sciences, University of Health Sciences, Lahore, Pakistan

**Keywords:** animal models, liver metastases, tumor progression, colorectal cancer, metastasis-related genes

## Abstract

Liver is the main target of colorectal cancer (CRC) metastasis. Currently, the number of reports is small, which describe changes in gene expression supporting liver metastasis. Here, a rat model was used for analyzing mRNA modulations during liver colonization and compared with available literature. In the model, CC531 rat CRC cells were injected *via* a mesenteric vein into isogenic WAG/Rij rats and re-isolated at early, intermediate, advanced, and terminal stages of liver colonization. These cells were used for RNA isolation. Microarrays were used for analyzing mRNA profiles of expression. The number of deregulated genes is comparatively large and only part of it has been studied so far. As reported to date, claudins and insulin-like growth factor-binding proteins (IGFBPs) were found to be deregulated. The fact that the chosen method is efficient is confirmed by the study of claudins and IGFBPs, which show altered expression in the initial stages of liver colonization and then return to normalcy. In addition, cadherin was described to be downregulated in epithelial–mesenchymal transition models. It can, therefore, be concluded that the models used are helpful in finding genes, which are instrumental for metastatic liver colonization.

## Introduction

With more than one million new cases, colorectal cancer (CRC) is one of the most common malignancies worldwide (1). In the primary operative treatment of CRC, metastasis is the limiting parameter. The progress of a CRC is also characterized by increased primary carcinoma growth and hematogenic and lymphatic spread. However, at the time of diagnosis, up to 25% of patients have a synchronous hematogenic metastasis, which is most frequently manifested in the liver. After resection of the primary tumor, a similar percentage (up to 25%) of the patients develops metastasis in the subsequent course of the disease, i.e., within the next 3 years (metachronous type of progression) (2–4). Surgery is only possible for a small proportion of these patients (about 10%). For the other patients, survival is limited to only 9–19 months (2–6).

When seeking explanations, why the liver is a main target of colorectal cancer metastasis, anatomical reasons are most often discussed. The liver represents the first capillary bed, in which disseminated colorectal cancer cells can become stuck. Subsequently, they grow and form life-threatening metastases, which are reason for the aggressive behavior and resulting mortality of CRC (5–7). Treatment of these metastases is rarely curative, if conventional surgery, radiotherapy, and chemotherapy are being used (8).

The primary tumors consist of a heterogeneous population of cells that are genetically distinct. This genetic variability allows the tumor cells to separate from the primary tumor and overcome various obstacles before growing in other organs. Nevertheless, only an extremely small part (0.001%) of disseminated tumor cells can form metastases (9, 10). This observation indicates that many aspects of the metastatic process are still unclear. Nevertheless, some of the sub-mechanisms are considered to be scientifically well explored. The metastatic process can be divided into three main processes, namely the initialization process, the progression process, and the establishment process. In order to develop a malignant and progressively metastasizing cell from a normal mucosal cell, many characteristics are necessary, which enable the cells to grow autonomously, continuously, and invasively (11, 12).

## Animal Models for Liver Metastasis

Typically, models should mimic the characteristics of the disease, which is to be investigated. Some animal models have been developed to mimic CRC and its progression. Most frequently, human tumor cells were transplanted subcutaneously into nude rodents (so-called xenografts), as the respective tumor growth in this model can easily be measured. However, the value of these models has been questioned, especially when it comes to assessing the efficacy of new drugs, because these tumors are normally non-invasive and do not form metastases.

Pending on the origin of tumor cells, transplantation models can be isogenic or xenograft models. In the case of isogenic models, usually mouse or rat tumor cell lines are used. In xenograft transplantation models, human tumor cells or human tumor pieces are injected and implanted into immune-incompetent (nude) animals. Orthotopic cancer models are based on the implantation of cancer cells into the organ, from which the tumor cells originated. In the majority of these models, however, tumor growth cannot be assessed by eye. With regard to xenografts, it was observed that the produced tumors are histologically a mixture of human tumor cells and murine stromal cells (13).

An example of a transplanted isogenic model is the rat colorectal cancer cell line CC531, which was originally developed from a colon cancer growing in a dimethyl hydrazine-induced WAG/Rij rat (14). This tumor grew in various organs, including lymph nodes, abdominal cavity, and liver (15). For a considerable time, this property was used to evaluate the efficacy and toxicity of new antineoplastic treatment modalities (e.g., drugs, irradiation, antibodies, photodynamic therapy, locoregional administration) in experimental liver metastasis (16–27).

However, this model suffered from its growth in organs, which could not be inspected regularly. Therefore, markers were introduced, which were to help in monitoring the growth of this tumor. Accordingly, CC531 cells were marked with genes that facilitate their detection, as well as their interaction with the environment. Examples of such marker genes are the *Escherichia coli* β-galactosidase (lacZ) gene (28). The exposure of cells, which are transfected with this gene, to X-Gal (5-Bromo-4-chloroindoxyl-β-d-galactopyranoside), leads to cleavage of this substrate into galactose and 5-bromo-4-chloro-indoxyl. The latter dye is air-dried to the blue dye 5,5-dibromo-4,4-dichloroindigo. The lacZ gene is considered a stable marker during tumor progression *in vivo* (28–37). Transfection of CC531 cells by the lacZ gene was performed by Wittmer et al. (38) and the resulting clone was used for determining the tumor load of the animals at the end of the respective experiments (39–45).

Green fluorescence protein (GFP) and its variants are also markers that allow the detection and sorting of tumor cells by using certain light wavelengths and fluorescence activated cell sorting (FACS) analysis, respectively (46–48).

Similar to the lacZ method, the luciferase reporter system is an alternative that enables an optical detection of tumor cells *in vitro* and *in vivo* (49, 50). In transfected tumor cells, the luciferase gene is stably expressed, resulting in the presence and activity of the luciferase enzyme. Exposure of these cells to the respective substrate (luciferin, coelenterazine) results in light emission, which can be directly measured and correlated to the size of the tumor (51). Both markers, enhanced GFP and luciferase, were introduced into CC531 cells to allow improved detection during the lifespan of the animals (47, 52).

This final model was used most recently to identify new genes that are involved in the early stage of rat liver metastasis (47, 52).

The respective experiments, detailing the re-isolation of CC531 cells, being stably transfected with GFP as well as luciferase genes, from rat liver at various stages of colonization are detailed in the subsequent review. The aim of these experiments was to describe the genetic characteristics of liver-metastasis as a self-regulating process, which has features that are independent from the primary tumor. So far, this question has not been sufficiently covered in the literature, although related work, which focused on the isolation of tumor nodules, was done by Velthuis et al. (44), Sun et al. (45), Georges et al. (53), and Speetjens et al. (54).

Specifically, the question was addressed, which temporal profile of gene expression tumor cells must show to enable their growth and metastasis in the liver. In view of the enormous genetic diversity of the primary tumor and the high number of disseminated tumor cells in the venous blood of carcinomas, this approach did not focus on cells obtainable by liquid biopsy, but used the liver as filter for those cells, which are able to form liver metastases. Consequently, the entire period of the metastatic colonization of the liver was investigated. It was hoped that the changes in gene expression detected in re-isolated tumor cells would be helpful in understanding the mechanism of action of liver colonization by CRC cells, as well as for finding a specific therapy.

## Preparation and Injection of CC531 Cells

Six- to eight-week-old male WAG/Rij rats with a body weight of 160–180 g were purchased from Charles River, Sulzfeld, Germany. The rats were kept and anesthetized as previously described (38, 47, 55). All animal experiments were approved by the responsible governmental animal ethics committee (Regierungspraesidium Karlsruhe, Germany). Logarithmically growing CC531 cells were prepared at a concentration of 4–8 × 10^6^ cells/500 μl depending on the experiment. After opening the abdomen, the cecum with its adjacent mesenteric vein was appropriately placed to allow the insertion of a 30G needle (BD, Heidelberg, Germany). Four hundred microliters of CC531 cell suspension was injected at a distance of ~1–1.5 cm from the cecum. The needle was gently inserted into the vein and the inoculation was administered slowly and lasted for 2–3 min, in order to achieve a good distribution of the cells in all liver lobes (Figures 1 and 2).

**Figure 1:** Schematic illustration of the injection site. The CC531 rat CRC cells were inoculated into the mesenteric vein to form liver metastasis.

**Figure 2:** Schematic illustration of the tumor cells’ isolation experiment. The CC531 rat CRC cells are injected into the rat liver and re-isolated after different time periods (3, 6, 9, 14, and 21 days). Cells isolated after 21 days were cultured for further 14 and 22 days *in vitro*. Proteins and mRNA were isolated from all cells for Western blot, as well as PCR and microarray, respectively.

## Re-Isolation of Hepatocytes, Kupffer Cells, and Tumor Cells from the Rat Liver

Ten rats (2 for each time point; i.e., 3, 6, 9, 14, and 21 days after tumor cell inoculation) were sacrificed and used for the experiment described below. It is also worth noting that all animals survived the experiment. An incision was made into the abdominal wall and the intestines were placed out of the abdominal cavity to locate the portal vein (Figure 1). The liver was washed and connection tissues were digested as described previously (47, 52, 53, 56). Subsequently, the liver was excised from the rat and placed into a sterile Petri dish. The liver was then treated with an appropriate enzyme cocktail (pronase and collagenase Type IV) and the resulting cell suspension of liver and tumor cells was transferred into tubes and layered carefully onto a Ficoll gradient medium. After centrifugation (15 min at 500 × *g*), hepatocytes, Kupffer cells, and tumor cells were obtained from the different layers of the interface (Figure 2). For better detection and to gain a high purity of isolated tumor cells, tumor cells were beforehand stably transfected with red fluorescence protein (RFP; Figure 3) and luciferase (Figure 4).

**Figure 3:** CC531 rat CRC cells re-isolated from rat liver after 6 days of tumor cells’ inoculation. **(A,B)** Microscopic photographs of CC531 cells after 5 and 30 h of their re-isolation from rat liver. Magnification ×200, the bars indicate a distance of 20 µm.

**Figure 4:** Light emission based on luciferase activity of CC531^RFP-LUC^ rat CRC cells, 5 × 10^5^ CC531^RFP-LUC^ cells were injected into the rat liver. Aspect after luciferin injection of tumor bearing animals. **(A)** 14 days following transplantation of CC531^RFP-LUC^ cells. **(B)** 21 days following transplantation of CC531^RFP-LUC^ cells. **(C)** 28 days following transplantation of CC531^RFP-LUC^ cells.

## Gene Expression Profile of the Re-Isolated Cells

From the genes analyzed by microarray, some genes, which were ≥2-fold up- or downregulated when compared to control cells, were chosen for subsequent analysis *in vitro* and in human CRC specimens.

### Claudins

The aim of this experiment was to determine changes in the expression profile of the CRC cells during their colonization of the rat liver in order to determine a specific, time-dependent modification of metastasis-relevant genes and processes for further studies. The mRNA of the re-isolated cells was used in cDNA microarrays to analyze the mRNA expression profiles of these cells during their growth in the rat liver. During liver colonization, claudins 1 and 4 showed two-phase changes in their expression, in correlation with their presumed function during liver colonization. Initially, a significant reduction in the expression of claudins (here: claudin 1 and claudin 4) was observed, which were up to eightfold reduced compared to the control (Table 1). To analyze whether this reduced expression is primarily due to contact with the new environment, a coculture of the tumor cells with isolated rat hepatocytes and Kupffer cells was carried out. However, no change in the expression of the affected claudins was observed. However, the expression of claudin 4 was increased when the shear and friction forces in the blood circulation were simulated experimentally. A reduction in the mRNA expression of claudins1 and 4 by siRNA caused a significantly increased migration and at the same time reduced the colony formation capacity of the tumor cells (*P* < 0.05), but had no effect on their proliferative capacity (47).

**Table 1:** Comparative expression of some genes, including adhesion molecules, insulin-like growth factor-binding proteins (IGFBPs), and chemokines.

Gene family/genes	Gene expression	Reference
**Adhesion molecules**		
*Cldn1*	Downregulated in early metastasis	(47)
*Cldn4*	Downregulated in early metastasis	(47)
*E-cadherin*	Downregulated in epithelial–mesenchymal transition (EMT)	(57–60)
**IGFBPs**		
*Igfbp3*	Upregulated in early metastasis	(52)
*Igfbp7*	Upregulated in early metastasis	(52)
**Chemokines**		
*Ccr1*	Upregulated in early metastasis	(61)
*Ccrl2*	Upregulated in early metastasis	(61)

An investigation of human CRC samples showed increased expression of claudins 1 and 4 by immunohistochemistry in stages I–III carcinomas, but at stage IV and in liver metastases, claudin expression was significantly reduced (*P* < 0.05). In addition, it was shown that an increased claudin 4 expression was correlated with a significantly reduced overall survival (log rank test, *P* = 0.018) (47).

### The Insulin-Like Growth Factor-Binding Proteins (IGFBPs) 3 and 7 Are Associated with Liver Metastasis of Colorectal Cancer

In a follow-up experiment, the family of IGFBPs was investigated more closely. Some members of this family also showed a highly significant change in their expression in the micro-array examination after re-isolation of CC531 rat CRC cells from rat liver. In contrast to the expression of the claudins, the expression of IGFBPs was initially significantly increased and normalized later, with the progressive infiltration of the liver by the tumor cells. IGFBP3 and 7, which represent the main group of IGFBPs and the side group of the related proteins, were selected from the group as a whole. A knockdown of both proteins resulted in reduced proliferation, colony formation, and migration (the latter only IGFBP3) of the CC531 cells.

In human tumor samples, expression of both genes was higher in UICC stages II and III than in stages I and IV. In addition, IGFBP3 was negatively correlated to the age of the affected patients in these samples and positively correlated with the expression of IGFBP7 (52).

### Role of Chemokines and Their Receptors in CRC Progression

The chemokines C-C chemokine receptor type 1 (CCR1) and C-C motif receptor-like 2 (CCRL2) are associated with colorectal cancer liver metastasis: The expression modulation of CCR1 and chemokine CCRL2 were investigated in the same rat liver metastasis model. In addition, their expression in rat and human CRC samples was also analyzed. In this experiment, we studied the effects of their knockdown on cellular properties in a panel of colorectal cancer cell lines. One rat and five human colorectal cancer cell lines were used for this purpose.

All cell lines were screened for mRNA expression of CCR1 and CCRL2 by reverse transcription polymerase chain reaction (RT-PCR). Cell lines with detectable expression were further investigated. Specifically, the cells’ proliferation, scratch closure, and colony formation was determined, respectively. Knockdown of the two genes resulted in modest but significant inhibition of proliferation (*P* < 0.05), scratch closure, and colony formation (*P* < 0.05).

The re-isolation of CC531 rat colorectal cells from rat livers after defined periods, followed by mRNA isolation, showed a clear modulation in the expression profile of these genes during the colonization process. In particular CCRL2 and CCR1 were upregulated 27 and 4 times, respectively, when compared with the control cells.

Finally, specimens from 50 patients with CRC were examined by quantitative RT-PCR for CCR1 and CCRL2 expression levels. All human CRC samples were positive for CCR1 and CCRL2 and showed a significant pairwise correlation (*P* < 0.0004), but there was no correlation with tumor stage or age of patients (61).

The chemokine receptor CCR5 was found to be increased in CC531 cells in a way similar to CCR1 and CCRL2. To investigate its importance, CCR5 (CD195) was blocked with the CCR5 receptor antagonist maraviroc in human colorectal carcinoma cells (SW480 and SW620). Subsequently, the effect of this blockade on the cell properties and the associated signal paths were examined. The blockade with maraviroc caused a significant proliferation inhibition and a marked arrest of the cells in phase G1 of the cell cycle. In addition, maraviroc caused a significant increase in apoptosis induction at the morphological level. Concomitantly, a significant modulation of several apoptosis-relevant genes was observed at the mRNA level and activation (posttranslational modification) of the caspases was observed at the protein level. The observations were depicted in a signaling pathway of CCR5, which summarizes the cytotoxic and apoptotic effects of maraviroc in colorectal carcinoma cells (62).

### The Regulation of Osteopontin and Functionally Associated Genes in the CC531 Model *In Vitro* and *In Vivo*

The expression of the matrix protein osteopontin, as well as that of osteopontin associated genes BSP II, Runx2, Hoxc8, MMP-7, and MMP-9 was also studied in CC531 cells during the colonization process and *in vitro*.

OPN, Runx2, and MMP-7 showed increased expression in the advanced stage of liver metastasis but subsequently showed reduced expression after the isolated tumor cells had been further cultured *in vitro*. In addition, an inverse regulation of Hoxc8, OPN, and Runx2 was observed. The cocultivation of the tumor cells with hepatocytes did not cause increased expression of OPN and RUNX2, whereas the addition of TGF-β1 induced overexpression of OPN and Runx2 in tumor cells but not in cocultured hepatocytes (52, 63).

## Discussion

The pathophysiologic consequences of gastrointestinal cancers’ metastases are a major cause of their mortality (2, 64, 65). After a large number of studies, tumors are genetically derived from heterogeneous cell aggregates (3, 66–68). Despite this genetic heterogeneity, individual disseminated tumor cells often follow the same pattern of metastasis formation. They grow initially in the liver, but not, or only in the further course, in other organs (10, 69, 70).

In addition, only a small fraction of the disseminated tumor cells succeed in forming metastases. In line with this, it must be borne in mind that disseminated tumor cells are not true metastases, but represent only tumor cells with a necessary but not sufficient precondition to metastasize. From their enormous number and high genetic heterogeneity/diversity, the real metastases are recruited (71).

One of the questions that have remained unanswered so far is what genetic characteristics these individual metastasis-producing cells have and how it is possible to identify them in the face of the enormous genetic diversity of the primary tumor and the large number of cells that separate from it? Morphological and genetic examinations of established metastases generally do not provide any clue since morphological aspects and genetic signatures differ only slightly in terms of mutations in tumor suppressor and oncogenes from the primary tumor (3).

Rather, identification of modulated gene expression, even if present for a short time only, would possibly allow inhibiting the metastasis process by means of targeted manipulations.

Therefore, the aim of this work was to analyze the literature regarding expression profiles of tumor cells during the entire period of metastatic colonization of the liver, in order to manipulate them in a targeted manner. For the main part of this review, a CRC tumor model was considered, which mimics the metastasis process. This model is based on CC531 rat -CRC cells, which were injected *via* the mesenteric vein into the liver of WAG/Rij rats and then re-isolated after various times (55). For an analysis of the genetic profile, a pure cell population is essential. In order to ensure this, two enrichment methods were used, i.e., a Ficoll gradient followed by FACS, which was based on the CC531 cells’ labeling with the marker protein RFP.

The mRNA expression profile of these cells was investigated during the entire liver-colonization process. Interestingly, genes were activated or deactivated at the beginning of the colonization process, and this alteration was related to the process progression.

With regard to the type of modulation, claudins and E-cadherin were found to be decreased, whereas the insulin-like growth factor binding proteins and chemokines showed increased expression. Notably, these modulations normalized later again.

For the claudins and E-cadherin, their diminished expression is an indication of the so-called epithelial–mesenchymal transition (EMT). This is in accord with the EMT theory, which states that in metastasizing tumor cells a phenotype change must first take place. These cells lose their adhesion properties and gain the ability to migrate. The loss of cell adhesion is caused, *inter alia*, by reduced expression of adhesion molecules such as claudines and E-cadherin (57–60).

During the colonization process, IGFBPs and chemokines showed a contrasting expression pattern (see Table 1).

## Conclusion

This review focusses on animal models, which identified genes that are modulated in their expression during liver colonization by CRC cells. The number of these genes is comparatively large and only a part of it has been identified so far. Nevertheless, the chosen method is efficient as is shown by the results on claudins, E-cadherin, insulin-like growth factor-related proteins, and chemokines, which show distinct modulation of expression during liver colonization. Such findings may contribute to exploiting the potential of these genes as suitable markers for early diagnosis or as targets of an effective therapy of liver metastasis.

## Author Contributions

HA is the main author. RG and AP have prepared the figures. MB reviewed the publication.

## Conflict of Interest Statement

The authors declare that the research was conducted in the absence of any commercial or financial relationships that could be construed as a potential conflict of interest. The reviewer, WW, and the handling editor declared their shared affiliation, and the handling editor states that the process nevertheless met the standards of a fair and objective review.
